The article "UIBVFED: Virtual facial expression dataset" was published in 2020. Journal: PLoS One.

# UIBVFED: Virtual facial expression dataset

**DOI:** 10.1371/journal.pone.0231266

**Published:** 2020-04-06

**Authors:** Miquel Mascaró Oliver, Esperança Amengual Alcover

**Affiliations:** Department of Mathematics and Computer Science, University of the Balearic Islands, Palma de Mallorca, Spain; National Institutes of Health, UNITED STATES

## Abstract

Facial expression classification requires large amounts of data to reflect the diversity of conditions in the real world. Public databases support research tasks providing researchers an appropriate work framework. However, often these databases do not focus on artistic creation. We developed an innovative facial expression dataset that can help both artists and researchers in the field of affective computing. This dataset can be managed interactively by an intuitive and easy to use software application. The dataset is composed of 640 facial images from 20 virtual characters each creating 32 facial expressions. The avatars represent 10 men and 10 women, aged between 20 and 80, from different ethnicities. Expressions are classified by the six universal expressions according to Gary Faigin classification.

## Introduction

Facial expressions are the most effective method for humans to express emotions; one emotion gives more information than a lot of words. Aware of this, artists looked for the most accurate way of representing facial expressions. Drawing manuals are visual references to solve this task [1]; [2]; [3]. For instance [4] presents a dataset that includes more than 2500 photographs classified by ages, shapes, sizes and ethnicities, each demonstrating a wide range of emotions.

The industry uses motion capture techniques (MOCAP) to achieve maximum realism. However, artists use traditional bibliographic research methods when MOCAPs are not an option, either for budget or for artistic concerns. To the best of our knowledge there is no any interactive software application to manage a database for facial expression description.

In the affective computing field public databases promote research into automatically detecting individual facial expression. Examples are the Extended Cohn-Kanade Dataset (CK+) [5], MMI [6], RU-FACS [7], Genki-4K [8], UNBC-McMaster [9], Multi-PIE [10], O’Toole [11], MAHNOB [12], and AMFED [13]. The latter includes a detailed description of the others. Kairos Web site [14] provides 60 facial databases to build face recognition. Face Recognition Web site [15] includes a list of 97 facial expression databases for the same purpose.

These databases differ in several aspects: images or videos captured in controlled environments; images or videos captured without any specific lighting or frame; real expressions versus feigned expressions; all types of expressions; or only joyful of pain expressions. Most of the expressions are labelled according to the Facial Action Coding System (FACS) [16] and none of these databases works with 3D avatars. Our goal is to develop an avatar dataset with the different facial expressions and emotional content. We aim to provide a tool more simple and agile than common bibliographic searching. Users will be able to select the character that better suites to their interests and produce a facial expression controlling the intensity in a very simple and interactive manner. Our dataset has to be suitably labelled according to the regular affective computing standards to support analysis and facial recognition methods validation. We offer a new working framework different to data in the wild and other controlled environments. The main advantage is that users will have absolute control of the scene to compare the data from less controlled environments.

Two tasks are needed to achieve this goal: design the avatars and produce the facial expressions. In the following sections we first introduce the preliminary work about avatar facial geometry, motion setup and expression categorization. Then we describe the method followed to implement UIBVFED. We also describe the process to produce the images stored in the dataset and the interactive application to manage them.

## Preliminary work

### Geometry and avatar configuration

With the experience of 20 years in 3D creation and training we conclude that avatar design and configuration for realistic facial expression is a very laborious task. Despite the research in the automation of this process [17]; [18]; [19], results are not widespread used. Moreover, the idea of creating an avatar dataset without a huge professional team would be innocent. Thus, we use software tools to support the process as exposed below.

There is no standard for facial geometry construction and animation. However, there is consensus about two desirable characteristics [20]. Firstly, *Edge loop* geometry to simulate muscular movement for facial motion to be similar to reality is recommendable. Secondly, *blendshapes* are the most effective way to represent facial action units. *Blendshapes* interpolate a number of points conveniently deformed as exposed in [20]; [21]. Depending on the desired precision, configurations can vary between 25 and 100 *blendshapes*. These deformations are often controlled with sliders in the software application. For an intuitive motion it is usual to create an animation *rig* to manage *blendshapes*. Although there is some research about *rigging* [22]; [17], there is no any *rig* definition standard.

Recently, the demand for avatar creation has increased due to the proliferation of independent productions, for instance videogames. Thus, big companies have created online Web sites to manage characters in a free and fast manner. Examples are Adobe with Mixamo [23] or Autodesk with Autodesk Character Generator [24]. The latter meets perfectly our needs. It allows the creation of two types of characters named *Premium* and *Standard*. The first includes 5 basic men and 5 basic women; the second includes 11 basic men and 11 basic women. Each character is customizable by editing some characteristics. Facial editable characteristics are the oval, eye sockets, ears, nose, cheeks, and the chin. This edition is possible blending the characteristics of 46 more characters defined in the application. It is also possible to customize the eye colour, skin, hair and other characteristics we are not interested in, such as clothing or the body shape. The result is a geometry file that can be downloaded with the option of choosing quads or triangles, different file formats (fbx, Unity fbx, Maya and 3DMax), 3 geometry definition levels, and bones facial motion (with less detail) or *blendshapes* (more precision).

Facial bones and blendshapes are the two classical alternatives for facial motion. Bones facial motion has two main advantatges over blendshapes. First, there is not any restriction on the number of labelled deformations. Instead, the user applies lineal rotation and translation transformations to the bones to deform the skin geometries. Second, it is not necessary to previously define a large set of deformations to later do interpolation among them. The only requirement is to define the points in the geometric mesh that will be affected by each bone and the degrees of freedom for each joint.

In our case, the disadvantages of blendshapes are not an issue since the Autodesk application automatically generates a large set of deformations for a specific facial motion. Additionally, labelled deformations from our system are easy to link with facial recognition tasks.

Both animation systems seamlessly integrate into Unity 3D development environment. Facial motion is simpler and more intuitive with blendshapes because deformation activation is done giving a specific value to the deformation intensity, whereas for bones you have to introduce translations or rotations in the space.

### Human emotion facial expressions

Among the reviewed literature Faigin [1] illustrates human facial expressions more exhaustively. This author provides a morphological analysis of facial characteristics grouped by areas: eyebrows, eyes, and mouth. He describes the muscular movement that an expression originates, analysing wrinkles, and looking for similarities with other morphologies. He considers a relevant number of photographs and other diverse artistic representations to typify each expression. The work concludes with a summary of all the expressions grouped into the six universal emotions (happiness, sadness, surprise, fear, disgust and anger) plus an additional group named “physical state expressions” that includes expressions for pain, effort, sleepiness, etc. 32 expressions describe the different facial morphologies. For instance six expressions describe sadness: (1) Crying: Open–mouthed; (2) Crying: Closed mouth; (3) Suppressed sadness; (4) Nearly Crying; (5) Miserable; (6) Sad.

## UIBVFED implementation

To implement the UIBVFED we considered maximum precision geometries that could be managed with Unity. We used *blendshapes* as facial motion technique. The goal was to develop a dataset and an application to deal with expressions interactively.

Each geometry file corresponds to a character and is formed by different group geometries. The skin group and the lower teeth geometries have facial motion *blendshapes*. The skin mesh group geometry is labelled *H_DDS_HiRes* and has 65 *blendshapes*. The lower teeth group geometry is labelled *h_Teeth_Down* and has 31 *blendshapes*. Each *blendshape* is characterized by a name which explains the deformation. Examples are *h_expressions*.*BMP_Up_h* for upper lip deformation for the B, M, and P sounds; *h_expressions*.*MouthOpen_h* for mouth opening; or *h_expressions*.*ReyeClose_h* for right eye closing. All facial deformations have values between 0 and 100 where 100 mean maximum deformation and 0 the absence of deformation.

We have used Autodesk Character Generator as a support tool to create 20 different characters, 10 men and 10 women, aged between 20 and 80 and different ethnicities as shown in Fig 1. These characters have been customized with this software tool. Therefore the UIBVFED software application allows the selection of the different characters, although it does not permit to change the predetermined configuration such as the age or the ethnicity.

**Fig 1:** UIBVFED characters in neutral position (without deformation).

We selected the suitable *blendshapes* for each expression. Then, we reproduced the expression using muscular movement descriptions and the sample images reported in [1]. Table 1 summarizes the values for each deformation for the sadness expression labelled as *Miserable*. The first column is the identification of the active *blendshape* and depends on the file order generated by the Autodesk application. The second column corresponds to the name. Finally, the third column is the deformation value. See the supplementary material for the complete list of the 32 expression values.

**Table 1:** *Blendshapes* for the sadness expression: *Miserable*.

Id	Blendshapes Exp: Miserable	Value
10	h_expressions.MPB_Up_h	50
21	h_expressions.JawCompress_h	50
32	h_expressions.RmouthSad_h	100
33	h_expressions.LmouthSad_h	100
36	h_expressions.Kiss_h	100
39	h_expressions.Chin_h	100
47	h_expressions.ReyeOpen_h	25
48	h_expressions.LeyeOpen_h	25
51	h_expressions.RlowLid_h	75
52	h_expressions.LlowLid_h	75
53	h_expressions.Rsad_h	100
54	h_expressions.Lsad_h	100

Fig 2 shows the application of these values to a particular character from our dataset.

**Fig 2:** Reproduction of the *Miserable* sadness expression on a character.

### Blendshapes versus facial action units

As mentioned before, tools to define expressions and standard codes to categorize them are critical. Rig systems are used to make *blendshapes* use more intuitive. However, from an artistic point of view the definition of expressions through action units has no interest. Nevertheless, if we want a dataset to be useful for expression recognition we need to compare *blendshapes* with the facial action units used in most databases.

To define this relation we only analysed those *blendshapes* that affect the character skin. This is because lower teeth blendshapes have the same name and, therefore, are redundant. For instance, for mouth opening the label *h_expressions*.*MouthOpen_h* is similar to *h_teeth*.*t_MouthOpen_h*. To analyse the correspondence between deformation and action units we compared one by one the *blendshapes* with the visual documentation available in (‘Facial Action Coding System (FACS)—A Visual Guidebook’ n.d.; FACS n.d.). The result of this analysis is an equivalency chart which is included as a supplementary material. The exact value of the blendshape geometric deformation (see column *Value* in Table 1) has been empirically adjusted to visually fit the FACS. From this chart we consider appropriate to highlight the following issues:

- There are some action units such as 1 (*Inner Brow Raiser*), 4 (*Brow Lowerer*), and 10 (*Upper Lip Raiser*) that can be reproduced by distinct *blendshapes*. These cases are more precise with *blendshapes* than with action units. Moreover, *blendshapes* distinguish between left and right.
- Action units that correspond exactly to their *blendshapes* are: 2, 5, 11, 12, 14, 16, 17, 18, 22, 27, and 44.
- Some action units can be reproduced combining several *blendshapes*. For example, action unit 9 (*Nose Wrinkler*) is the combination of *LipUp* and *LbrowDown* (without wrinkles), and action unit 13 (*Cheek Puffer*) is the combination of *SmileClose* and *JawCompress*.
- Some *blendshapes* individually serve for different action units. Examples are *MouthOpen* that represents unit 25 (*Lips part*) and 26 (*Jaw drop*), or *eyeClose* that represents units 41, 42, and 43 for different grades of closed eyes.
- The majority of *blendshapes* that are used for talking animation are not codified as unit actions. Likewise unit actions for eyes and head movement do not have their corresponding *blendshapes*. This is because these motions in particular are done separately from skin deformation. More specifically eye movement and neck torsion are done with skeletal animation techniques.

### Dataset implementation

For the implementation of the UIBVFED dataset we used the videogame engine Unity [25] that allows to manage geometry file deformations for any facial expression. We created a data structure that contains the character set and the two group geometries with deformations for each character.

More specifically, our dataset allows the activation of the 32 facial expressions according to [1]. Characters are presented on an empty Unity scene on a white background and a basic lightening with three light points. It is only possible to see a character at once.

To create the dataset we generated the 32 facial expressions for each one of the characters. We captured an image for each expression with a frontal camera. Registered images were grouped into the universal emotions and labelled with the character name and the expression name following the same terminology as in the literature [1]. All images have a resolution of 750 x 133 pixels and are saved in png format.

We also developed a software application to interactively visualize the expressions. The application allows manual selection of the character and the facial expression, turn on and turn off the expression, character rotation, zoom in and zoom out. It is accessible through a browser compatible with WebGl technology Fig 3 shows the application graphical user interface with all the features.

**Fig 3:** UIBVFED application GUI.

As before mentioned, all avatars share the same blendshapes names. Therefore, assigning the different expressions to the characters is easy.

We have developed two applications with Unity 3D: one to build the database and another to build the interactive interface. The first application selects the characters one by one, activates all blendshapes for each expression and stores the image. The second, increments the blendshape value from zero to a maximum value (see Table 1) for each time increment. This is done while the user is holding key 1. By doing so the user is able to visually control the intensity of the expression.

Fig 4 shows the reproduction of the *Laughter* expression on a six different characters with the same intensity value.

**Fig 4:** Reproduction of the *Laughter* expression on a six different characters.

### Facial landmarks

As exposed in [26] in facial recognition all methods and techniques include a feature extraction process. To identify the face oval, eyebrows, eyes, nose and mouth different methods are used. These methods place a set of landmarks over the face image. One of the most cited is [27].

UIBVFED dataset was extended with the landmarks that correspond to 51 points in the 3D space to facilitate expression recognition. These points define the character morphology and its expressions as in the example shown in Fig 5.

**Fig 5:** *Enraged Shouting* expression with landmarks.

We placed landmark points following the 51 points model similar to the one proposed in [28] which empirically demonstrated the best results. These points were distributed on the basis of an index of the character mesh vertices. Although geometry can be different, configuration among characters is similar and therefore landmarks can be equally placed. There is only one case of a character with eyebrow points under the correct place, but with the same morphology. This is because eyebrows are represented with texture that in this particular case remains displaced. Since the morphology is correct, there should be no problem for expression recognition.

In the dataset each expression has an image with and without landmarks. A text file for each character with the data on the 51 points for each facial expression is also included. Expressions are ordered according to [1] and landmarks according to [28]. All characters have the same height and are located at the origin of the space.

## Conclusions

This work is oriented to multidisciplinary areas that could benefit from facial expression virtual prototyping. We offer a 3D avatar expression dataset to the research community.

After this work we can conclude the following:

1. The dataset presented in this work is the first 3D avatar expression dataset based on virtual characters. Additionally, it is the first and the only one labelled according to the 32 types of expressions defined by Faigin which implies a better precision than the other datasets found in the literature.
2. The dataset together with the software application that allows to interactively manage the expressions are a more easy to use and intuitive tool than the other available tools, both for traditional artists or 3D creators that want to represent facial expressions without using MOCAP techniques.
3. The UIBVFED dataset is a new tool for emotion and expression recognition validation. All the expressions are based on *blendshapes* as a new artistic point of view and are conveniently labelled according to unit action standard criteria. The dataset contains the landmarks in 3D space to support the research tasks based on landmark interpretation. More explicitly, our database can be useful to prove the goodness of other methods for landmark generation. In addition it simplifies the expression extraction process by offering geometrically fixed landmarks.

We believe that our contribution represents a new approach that enhances human emotion representation and could open new research frontiers. One possible criticism to our system is that all characters use the same blendshape deformation value for a specific expression. Obviously this can be seen as an inaccuracy. In reality the intensity of an expression for each individual depends on different psychological or physiological parameters that our system cannot reflect. However, the resemblance among characters with the same expression is mitigated by the differences among the facial geometries topology for each character. As future work we could consider six distinct proposals:

- Introduce small random variations of the maximum deformation values.
- Allow the storage of images interactively, giving the intensity control to the user.
- Add a new video generation option to the interactive application.
- Expand the number of characters including children and teenagers.
- Allow data generation relying on the expression intensity.
- Create files with geometry information for 3D printing.

## Supporting information

S1 Data List of blendshapes. (ODS)

S1 Video Facial expression interactive application video. (MOV)
